# An Image Recognition Framework for Oral Cancer Cells

This article has been retracted.

**DOI:** 10.1155/2021/2449128

**Published:** 2021-10-14

**Authors:** Hao Zhang, Wei Li, Hanzhong Zhang

**Affiliations:** ^1^Department of Stomatology, The Central Hospital of Wuhan, Tongji Medical College, Huazhong University of Science and Technology, Wuhan 430014, China; ^2^Huazhong University of Science and Technology, Wuhan 430014, China

## Abstract

Oral squamous cell carcinoma (OSCC) is a common type of cancer of the oral cavity. Despite their great impact on mortality, sufficient screening techniques for early diagnosis of OSCC often lack accuracy and thus OSCCs are mostly diagnosed at a late stage. Early detection and accurate recognition of OSCCs would lead to an improved curative result and a reduction in recurrence rates after surgical treatment. The introduction of image recognition technology into the doctor's diagnosis process can significantly improve cancer diagnosis, reduce individual differences, and effectively assist doctors in making the correct diagnosis of the disease. The objective of this study was to assess the precision and robustness of a deep learning-based method to automatically identify the extent of cancer on digitized oral images. We present a new method that employs different variants of convolutional neural network (CNN) for detecting cancer in oral cells. Our approach involves training the classifier on different images from the imageNet dataset and then independently validating on different cancer cells. The image is segmented using multiscale morphology methods to prepare for cell feature analysis and extraction. The method of morphological edge detection is used to more accurately extract the target, cell area, perimeter, and other multidimensional features followed by classification through CNN. For all five variants of CNN, namely, VGG16, VGG19, InceptionV3, InceptionResNetV2, and Xception, the train and value losses are less than 6%. Experimental results show that the method can be an effective tool for OSCC diagnosis.

## 1. Introduction

With the development of modern society, the incidence of oral cancer is increasing year by year in the world. The latest worldwide census showed that malignant tumors of the oral cavity and throat accounted for sixth place among all neoplastic lesions [1]. As a fatal disease, oral cancer [2] has a 5-year survival rate of only 30–40% (lip cancer can reach 80%) [3]. Owing to the continuous efforts of professionals, modern oral malignant tumor treatment technology has been dramatically improved [4]. Still, in terms of the survival rate of such patients, there has been no significant improvement in the past few decades. This is mainly due to the lack of general understanding of oral cancer, leading to early oral cancer often failing to attract enough attention from patients and delaying the best treatment opportunity, resulting in irreversible consequences. Therefore, the early detection, prevention, and treatment of oral diseases, especially oral cancer, are important for improving the cure rate of cancer and curing the tumor [5].

In the pathological diagnosis of cancer tumors, it is common to observe and qualitatively describe cell morphology. The primary method to investigate cell morphology is to keep ultrathin sections under a microscope and examine cell structures. However, this traditional analysis method is mainly based on a large number of observations and qualitative descriptions [6]. On the one hand, this method requires a large amount of inspection work and provides low inspection efficiency. It can also lead to misidentification and affect the accurate diagnosis of the disease. On the other hand, the analysis and recognition of pathological images are limited by the doctor's experience and visual resolution of images [7]. It is easy to produce subjective factors and lacks a scientific and objective quantitative basis.

Digital image processing [8] refers to using digital computers and other related digital techniques to apply certain operations and processing to images to achieve a specific intended purpose. For example, to make faded photos clear, extract meaningful cell features from medical micrographs, and so on, digital image processing can be divided into several aspects: image digitization, image information storage, image information processing, image information output, and display [9].

The acquisition of image information in digital image processing is the study of how to represent an image as a set of numbers (digital photos) and input them into a computer or digital device for analysis and processing. This image conversion process is called digitization [10]. At each pixel location of the image, the image's brightness is sampled and quantized to obtain an integer value representing its brightness and darkness on the corresponding point of the image [11]. After the conversion is completed for all pixels, the image is represented as an integer matrix as the object of computer processing. In an image, each pixel has two attributes: position and grayscale. The position is determined by the sampling point coordinates in the scan line, also called row and column, and the integer that represents the brightness and darkness of the pixel position is called grayscale. The most commonly used digital instruments for processing images are digital cameras, flying spot scanners, and microdensitometers.

Digital pathology is the process of digitization of tissue images and slides. This process of digitization could enable more efficient storage, visualization, and pathologic analysis of tissue and could potentially improve the overall efficiency of routine diagnostic pathology workflow. The main processing techniques for cancer cell digital pathology include effective preprocessing, image segmentation, feature extraction, and classification methods. It is based on the morphology, structure, texture, and other characteristics of the cells reflected in the pathological pictures under the microscope to determine the standard for determining benign and malignant tumors to distinguish the cancer cells from the normal cells [12]. Extracting effective feature parameters and improving the recognition rate is the focus of cell digital image processing. In the analysis of microscopic cell images [13], mathematical morphology [14] is one of the commonly used methods. Mathematical morphology is suitable for digital image analysis. It is easy to obtain information such as the size, shape, direction, and connectivity of the target, which can extract morphological features. The effect of opening and closing operations to cut peaks and fill valleys is very suitable for denoising and segmentation cell images.

The rest of the paper is ordered as follows. In Section 2, different oral cancer recognition methods are described.  Section 3 provides a detailed discussion of the proposed method. The results are presented in Section 4 and the conclusion is given in Section 5.

## 2. Related Works

With the development of quantitative image analysis and the advent of image recognition techniques and its wide application in medical diagnosis, pathology has produced a new branch of computer image recognition research [15]. The image recognition techniques are introduced into the doctor's diagnosis process. Computer image analysis and recognition technology are used to study the characteristics of pathological morphology and structure of related tissues and discuss its application in diagnosis, classification, and prognosis judgment [16]. Image processing techniques can improve the recognition accuracy rate and reduce the labor intensity and workload of the person, eliminate the misdiagnosis and missed diagnosis caused by the psychological adaptability of manual detection and fatigue, and assist the doctor in making the correct diagnosis to a considerable extent.

Recently, with the gradual development of computerized tumor pathology recognition technology, foreign experts have pointed out the limitations of selecting fixed thresholds when extracting units from complex irregular backgrounds in the segmentation of pathological microscopic images and proposed the threshold theory of change which has achieved good results. German experts proposed a binary spatial organization classification method [17] in 2003, using stochastic geometric processes for nonlinear deterministic analysis and artificial neural networks (ANN) to assist in diagnosing breast cancer, pancreatic cancer, and prostate cancer and a series of prominent results have been achieved.

In terms of products, the Image-Pro Plus [18] developed by US Media Cybernetics is an entire 32-bit image processing and analysis system software that represents the latest international level. The software is suitable for professional image processing systems in medicine, scientific research, industry, and other fields. However, because it is a general-purpose commercial software, it can only provide corresponding data indicators for doctors' reference.

In recent years, the artificial neural network expert diagnosis system has become a research hotspot at home and abroad. The application of this technology in the field of stomatology has also achieved better results. Hung et al. [19] used an artificial neural network to predict the incidence of oral cancer in high-risk populations. In this study, 2027 adults received a questionnaire about smoking, drinking, and other bad habits and a professional dentist's examination to determine their final diagnosis. The data of 1,662 adults were used as training data into the 3-layer feed-forward backpropagation neural network, and the data of the remaining 365 people were used to test the effectiveness of the trained neural network. The sensitivity and specificity of manual screening were 74% and 99%, respectively, while the sensitivity and specificity of neural network detection results were 80% and 77%, respectively. Therefore, the higher sensitivity of the neural network used in screening high-risk groups of oral cancer has certain practical value. Still, its low specificity needs to be further studied to reduce the false-positive rate. In 2005, Campisi et al. [20] applied fuzzy neural networks to study cytokine expression in oral cancer and precancerous lesions. It detected the expression of BCL-2, survivin, and proliferating cell nuclear antigen in the lesions of 8 human papillomavirus-positive oral leukoplakia patients and applied a fuzzy neural network to determine the correlation between the cytokines as mentioned earlier and human papillomavirus infection. The results showed that survivin is related to the expression of proliferating cell nuclear antigen (PCNA) and human papillomavirus infection in leukoplakia lesions. In addition, the fuzzy neural network can be used as a credible and highly accurate research tool in the research of a small sample size. Jaremenko et al. [21] proposed an automatic image recognition method based on Confocal Laser Endomicroscopy images of the oral cavity, using the traditional pattern recognition methods with several local binary patterns, and histogram statistics and used random forest (RF) and support vector machine (SVM) for the classification. Rodner et al. [22] showed that segmentation-based image recognition has the potential to be applied to cancer recognition in Confocal Laser Endomicroscopy images of the head and neck region. Tanriver et al. [23] explored the applications of image processing techniques in the detection of oral cancer. A two-stage deep learning model was proposed to detect oral cancer and classify the detected region into three types of benign, oral potentially malignant disorders carcinoma with a second-stage classifier network. Kim et al. [24] developed a survival prediction method based on deep learning for oral squamous cell carcinoma (SCC) patients and validated its performance. The proposed method was compared with random survival forest (RSF) and the Cox proportional hazard model (CPH) and the proposed model showed the best performance among the three models. Tseng et al. [25] applied machine learning for oral cancer prediction 674 patients. Although the method ignored the time element, it was based on the major oral cancer patient dataset to date and is a prominent early effort to apply machine learning to oral cancer survival prediction.

In this study, an image recognition model is developed for the accurate prediction of oral cancer. Morphological analysis and calculation were performed on the segmented cell regions using machine learning techniques such as convolution neural network to extract distinct and prominent features of the cancer cells followed by prediction of cancer in these cells. Experimental results show that the proposed technique is effective in the prediction of cancer and can be an effective tool for the diagnosis of oral cancer.

## 3. Methodology

### 3.1. Classification and Recognition of Cancer Cell Images

Image segmentation refers to the process of dividing an image into regions with various characteristics and extracting the target of interest. It is a key step of image processing and further image analysis. It is a low-level computation technique and the most basic and important research process in computer vision. The quality of image segmentation results directly affects the quality of subsequent analysis, recognition, and interpretation. Based on an efficient image segmentation technique, feature extraction and parameter measurement of the target image can be performed, making higher-level image analysis. Therefore, the research on image segmentation is of great significance in the field of image processing. In this article, the main morphological characteristics of the nucleus of the cells are used to determine whether the cell is malignant or normal. Therefore, the primary problem of cancer cell identification is to separate the nucleus from the background through segmentation and process and identify the nucleus.

We use the concept of a set to give the following definition of image segmentation:

Let the set *R* represent the entire area of the image, and the segmentation of *R* can be accomplished by dividing *R* into *N* nonempty subsets. The subregion can be represented as *R*_1_,  *R*_2_,  *R*_3_,…,  *R*_*N*_.

Suppose a given uniformity measure *P* is a binary logic function. If a certain area meets a certain uniformity, its *P* value is TRUE; otherwise, it is FALSE. These *N* nonempty subsets satisfy the following five conditions given in Table 1.

The above conditions not only define segmentation but also guide how to perform segmentation. The image segmentation is always carried out according to some segmentation criteria. Condition 1 and Condition 2 indicate that the correct segmentation criteria should be applicable to all regions and all pixels, while Condition 3 and Condition 4 indicate that reasonable segmentation criteria should help determine the representative features of pixels in each image region, and Condition 5 indicates complete segmentation. The criteria should directly or indirectly have certain requirements or restrictions on the connectivity of pixels in the area.

After removing the image noise, the integrity and connectivity of the target are well maintained. At this time, the microscopic cell image only has two parts: the background and the nucleus, and the gray values of these two parts are quite different. The target can be segmented with a relatively simple threshold segmentation method, and the objective is to effectively determine the threshold. There are many threshold segmentation methods; this study uses the most typical maximum between-class variance threshold method. The basic principle is to divide the image histogram into two groups at a certain threshold and determine the threshold when the variance between the divided two groups takes the maximum value. The algorithm is briefly introduced below (*k* is the threshold).

Using the steps of Algorithm 1, the result of image segmentation can be obtained as shown in Figure 1. We can see that the processed image maintains the basic shape of the nucleus target, and the nucleus is extracted by an automatic threshold. After removal, the suspicious cell nucleus can be extracted more accurately.

The normal nucleus, cytoplasm, and cytoplasm background are all treated as nontarget areas and discarded. Suspicious nuclei and cell clusters are better preserved, but there are a few holes in the preserved area. The following will simply fill in the cavity to facilitate the individual processing of the cell nucleus and extract appropriate characteristic parameters.

To completely extract the nucleus and accurately calculate the parameters, these holes need to be filled. We employ the black area principle to fill the voids in the core. The specific method is to first binarize the image and then perform the inverse processing so that the original hollow area becomes black, and the nucleated area becomes white. The area of the black area in the inverted image is calculated due to the hole. Since the area is generally very small, we can select the area threshold CS (the number of pixels). When the area of the black area is smaller than CS, we can save the area and finally make the saved area similar in the backup image with holes Color filling. Similar colors are selected based on empirical values so that the cell nucleus is more completely approximate to its original shape. After the experiment, the value of Cs is 200. The filling result obtained is shown in Figure 2.

### 3.2. Deep Learning Model

Deep learning is a type of machine learning, and machine learning is the necessary path to realize artificial intelligence. Deep learning technology is widely used in tasks such as image and speech processing. Traditional machine learning methods use extract image features using Global feature descriptors such as histograms of oriented gradients, local binary patterns, and color histograms. These are hand-crafted features that require domain-level expertise. Instead of using hand-crafted features, deep neural networks implicitly extract features from images in a hierarchical manner. Lower layers learn low-level features such as edges and corners, whereas middle layers learn color, shape, and so on and higher layers learn high-level features representing the object in the image.

Among the deep neural networks, the convolutional neural network is the most famous network structure for processing images in deep learning. A convolutional neural network (CNN) can characterize learning and can classify input information according to its hierarchical structure, so it is also called a “translation-invariant artificial neural network.” We employed the different models of CNN for image prediction such as Visual Geometry Group with 16 layers (VGG16), VGG19, InceptionV3, Xception, and Inception_resnet_v2. VGGNet is one of the earlier batches of excellent neural networks. VGGNet was originally used to analyze and compare ovarian cancer images with AlexNet, GoogLeNet, and so on and a new network was proposed with higher accuracy on this basis [25]. It shows the feasibility of this model for cancer-related image recognition. In this study, we employed CNN for oral cancer cell recognition. The proposed VGG convolutional neural network model is composed of 13 layers of convolutional layers and 3 layers of fully connected layers. There are three main features, small convolution kernel, small pooling kernel, and fully connected transconvolution. The required input image data size is 224 × 224 × 3, which has fewer parameters and reduces the complexity of the model. The multilayer convolution structure can perform more nonlinear transformations than a single convolution layer, which is conducive to extracting high-level image features. Not only is InceptionV3 a well-known network of CNN, but also it has been used many times in the intelligent recognition research of other cancers. InceptionV3 consists of 5 convolutional layers, 3 pooling layers, 1 fully connected layer, and 11 Inception Module compositions. InceptionV3 has three main features; first, it uses different sizes of convolution kernels, which can extract different features and fuse them. The second pair of different sizes of convolution kernels use different padding to make the output feature map. The third convolution is used for the fusion of different channels of the feature map. The core idea is to increase the depth and width of the network to improve the performance of the CNN network and to avoid excessive loss of extracted image features. InceptionV3 solves the shortcomings of the VGG series well. InceptionV3 widens the network and uses different sizes of convolution kernels to deconvolve it.

Both ResNet and Xception are well-known networks in the field of deep learning and are widely used in the detection, segmentation, recognition, and other fields. ResNet is a residual network model with excellent performance. It constructs a deep neural network through residual connections, which can avoid gradient disappearance and gradient explosion caused by deep connections, and can effectively solve the situation that the accuracy rate tends to be flat in the later stage of training, but the training error becomes larger. Xception is a CNN architecture based entirely on deeply separable convolutional layers. Since its architecture is a linear stack of deeply separable convolutional layers with residual connections, the architecture is more convenient in definition and modification. InceptionResNetV2 is an early modification of the InceptionV3 model and is combined with some ideas of ResNet due to the existence of shortcuts in its model, deeper networks can be trained, and the Inception module can be simplified. The accuracy of this model is more advantageous than InceptionV3, ResNet152, and so on.

## 4. Experimental Results

Since the current database for oral cancer recognition does not have a more complete or authoritative version, to better provide a benchmark for the study of this problem, this article has enhanced the data of a similar project database on GitHub [26] and used it as the project's dataset. The original dataset sample includes two categories of images: normal and cancerous. In the original dataset, Class0 is a normal oral sample image, and the number before data enhancement is 150. Class1 is a diseased oral cancer sample image, and the number before data enhancement is 25. Figures 3 and 4 show normal and diseased images of oral cells samples. It can be observed that the two types of images show nearly similar patterns when observed through the naked eye. Therefore, it is more important to use intelligent assisted diagnosis methods to differentiate normal and diseased images.

In this experiment, we employed a pretrained network on the imageNet dataset for migration learning, followed by several layers of fully connected layers. Transfer learning is a machine learning method that transfers knowledge in one field to another field so that the target field can achieve better learning results. Since the deep learning model requires a large amount of training set data support, this experiment uses the method of transfer learning to make up for the lack of the number of training sets to improve the accuracy of the results.

In this experiment, the activation function used for the proposed CNN in the fully connected layer is rectifier linear unit (ReLU), the number of neurons in the final classification layer is 2, and the softmax activation function is used. ReLU for short is a piecewise linear function that will output the input directly if it is positive; otherwise, it will output zero. In this experiment, the weights pretrained on ImageNet have been frozen, no longer participate in the changes in neuron values caused by subsequent training, and only train the newly added fully connected layer. The activation function is used because the activation function introduces nonlinear characteristics into the network so that the neural network can be applied to many nonlinear models.

Next, we employed the Learning Rate Scheduler to dynamically adjust the learning rate to cope with the gradual reduction of the required step size as the number of training rounds increases. The input is a function, the input of the function is the current epoch number, and the return is the corresponding learning rate. In addition, this experiment also sets ReduceLROnPlateau to dynamically reduce the learning rate when the training is stagnant to avoid the phenomenon that the excessively high learning rate oscillates near the optimal solution. We selected the “Adam” optimizer, “categorical_crossentropy” loss function, and 50 epochs. The training results of the six models are shown in Figures 5–9 for VGG16, VGG19, InceptionV3, InceptionResNetV2, and Xception, respectively.

## 5. Conclusion

It can be observed in Figures 5–9 that the two losses (loss and val_loss) are decreasing and the two acc (acc and val_acc) are increasing. For all the five models of VGG16, VGG19, InceptionV3, InceptionResNetV2, and Xception, the train and value losses are less than 6%, so this indicates the modeling is trained in a good way. The val_acc is the measure of how good the predictions of a model are. In this paper, the model we proposed was trained pretty well after 50 epochs, while the rest training is not necessary.

## Figures and Tables

**Figure 1:** The result after segmentation.

**Figure 2:** Filled result.

**Figure 3:** Normal image samples.

**Figure 4:** Diseased image samples.

**Figure 5:** VGG19 training result.

**Figure 6:** VGG16 training result.

**Figure 7:** InceptionV3 training result.

**Figure 8:** InceptionResNetV2 training result.

**Figure 9:** Xception training result.

**Algorithm 1:** Variance calculation.

**Table 1:** Uniformity measure conditions.

1.	∪_*i*=1_^*N*^*R*_*i*_=*R*, *R*_*i*_ ≠ *ϕ*
2.	*R*_*i*_∩*R*_*j*_=*ϕ* *i* ≠ *j*
3.	*P*(*R*_*i*_)=TRUE *i*=1,2,…*N*
4.	*P*(*R*_*i*_ ∪ *R*_*j*_)=FALSE *i* ≠ *j*
5.	*R*_*i*_ is the connected region, *i*=1,2,…*N*.

## Data Availability

The datasets used and analyzed during the current study are available from the corresponding author upon reasonable request.
